This article has been retracted.

# Mild Hypothermia Promotes Ischemic Tolerance and Survival of Neural Stem Cell Grafts by Enhancing Global SUMOylation

**DOI:** 10.1155/2022/6503504

**Published:** 2022-05-27

**Authors:** Heng Cai, Xiaofang Ma, Dading Lu, Liangyu Chen, Xiyun Bian, Nan Zhang, Wei Tang, Xiaozhi Liu, Zhiqing Li

**Affiliations:** ^1^Department of Neurosurgery, Shengjing Hospital of China Medical University, Shenyang 110004, China; ^2^Liaoning Clinical Medical Research Center in Nervous System Disease, Shenyang 110004, China; ^3^Key Laboratory of Neuro-oncology in Liaoning Province, Shenyang 110004, China; ^4^Central Laboratory, The Fifth Central Hospital of Tianjin, Tianjin 300450, China; ^5^Tianjin Key Laboratory of Epigenetics for Organ Development of Preterm Infants, The Fifth Central Hospital of Tianjin, Tianjin 300450, China

## Abstract

Cerebral infarct penumbra due to hypoxia and toxin accumulation is not conducive to the transplantation of neural stem cells (NSCs), although mild hypothermia can improve the local microenvironment of the ischemic penumbra and exert neuroprotective effects. However, insufficient understanding of the molecular mechanism by which mild hypothermia protects the brain limits widespread clinical application. This study evaluated the molecular mechanism of mild hypothermia-induced brain protection from the perspective of global protein small ubiquitin-like modifier (SUMO) modification, with the aim of improving NSC transplant survival rates in the penumbra to enhance neurological function. NSCs from neonatal rats were extracted to detect the effects of hypoxia and mild hypothermia on SUMOylation modification levels, cell stemness, and hypoxia-induced injury. Overexpression and knockdown of UBC9 in NSCs were used to evaluate their ability to maintain stemness and withstand hypoxic injury. Finally, a rat middle cerebral artery occlusion (MCAO) model was used to verify the effect of mild hypothermia treatment and UBC9 overexpression on neural function of NSCs following penumbra transplantation in rats. Results showed that hypoxia and mild hypothermia promoted both the SUMOylation modification and maintenance of NSC stemness. Overexpression of UBC9 enhanced the abilities of NSCs to maintain stemness and resist hypoxic injury, while UBC9 knockdown had the opposite effect. Following transplantation into the ischemic penumbra of MCAO model rats, mild hypothermia and *Ubc9*-overexpressing NSCs significantly reduced cerebral infarct areas and improved neurological function. In conclusion, this study demonstrated that global protein SUMOylation is an important molecular mechanism for NSCs to tolerate hypoxia, and mild hypothermia can further increase the degree of global SUMOylation to enhance the hypoxia tolerance of NSCs, which increases their survival during transplantation in situ and ability to perform nerve repair in the penumbra of cerebral infarction.

## 1. Introduction

China ranks first in the world for the number of people experiencing stroke and, with the advent of an aging population, this trend is increasing annually [1–3]. According to reports, the prevalence of ischemic stroke in China was 1981 per 100,000 in 2017, with a mortality rate of 149 per 100,000 [2], thus imposing a heavy burden on families and society. Current treatment measures for cerebral infarction involve basic support and monitoring, dehydration to reduce intracranial pressure, anticoagulation, scavenging of free radicals, and nourishing nerves in an attempt to prevent complications and reduce mortality [4, 5]; however, the efficacy of all these methods remains uncertain. Therefore, in clinical practice, the implementation of an effective treatment plan is particularly important for improving the survival of patients and their quality of life.

In recent years, NSCs have yielded high hopes for the treatment of stroke, especially ischemic cerebrovascular disease [6]. Theoretically, NSCs transplanted into the penumbra at the edge of cerebral infarction will proliferate for a few generations and then differentiate to supplement neurons and glial cells, thereby repairing damage and improving nerve function. However, in fact, the penumbra microenvironment exhibits severe hypoxia and accumulation of large amounts of toxic substances that are extremely unfavorable for the local survival of transplanted NSCs, which severely limits their application. Therefore, improving the survival of transplanted NSCs in the penumbra is key for the treatment of ischemic cerebrovascular disease.

Nowadays, the application of mild hypothermia for brain protection has attracted increasing attention and gradually been implemented in clinical practice. A large number of international trials have confirmed the effectiveness and practicability of mild hypothermia in clinical applications, which can reduce the mortality rate and effectively improve the quality-of-life of patients with ischemic cerebrovascular disease [7–9]. However, as most reports only describe the clinical efficacy and methods of mild hypothermia treatment, the exact mechanism of its action has not been clarified. This restricts its wide acceptance by doctors and, to a certain extent, widespread promotion in clinical practice. Therefore, it is necessary to have a deeper and comprehensive understanding of the molecular mechanism by which mild hypothermia protects the brain to help doctors provide more precise treatment plans for patients with cerebral ischemia.

Small ubiquitin-like modifier- (SUMO-) mediated SUMOylation, a form of posttranslational modification of proteins, is used by cells to respond to external stress and adapt to changes in the internal environment [10]. SUMO modification of proteins requires the cascade reaction of SUMO activating enzyme (E1), conjugating enzyme (E2 and UBC9), and ligase enzyme (E3) [11–13]. Neurons can reportedly antagonize the adverse microenvironment of hypoxia by increasing global SUMOylation of a large number of proteins, such as hypoxia-inducible factor 1*α* (HIF-1*α*), and mild hypothermia can further increase global SUMOylation in neurons [14–16]. Indeed, this enriches the molecular mechanism underlying mild hypothermia-induced brain protection to a certain extent. At present, no reports describe the effects of hypoxia and mild hypothermia on protein SUMOylation in neural stem cells (NSCs). Moreover, it is unknown whether transplantation of NSCs overexpressing SUMO into the edge of a cerebral infarction, with or without mild hypothermia, can increase the survival rate of NSC grafts and improve prognosis.

Therefore, this study investigated the effects of hypoxia and mild hypothermia on global SUMOylation of NSCs, as well as their proliferation, differentiation, and hypoxia tolerance. We also transplanted NSCs overexpressing UBC9 into the cerebral ischemic penumbra of a rat middle cerebral artery occlusion (MCAO) model to evaluate their survival *in vivo*, as well as effects on the neurological functions of rats. In summary, the results show that mild hypothermia can promote the ischemic tolerance and survival of NSC grafts by enhancing global SUMOylation and improve the neurological function of rats. These conclusions identify a molecular mechanism supporting the brain protection elicited by mild hypothermia and provide a guide for increasing the survival of NSC grafts to improve the prognosis of patients with cerebral infarction.

## 2. Materials and Methods

The research conforms to NIH (2011) *Guide for the Care and Use of Laboratory Animals* (8th Edition, Institute for Laboratory Animal Research, Division on Earth and Life Studies, National Research Council of the National Academies Press).

### 2.1. Experimental Rats

Total number of 60 12-week-old male and 5 new-born (within 1 day) female Sprague-Dawley rats were purchased from SPF Biotechnology Co., Ltd. (Beijing, China). These rats were housed in the Animal Experimental Center of the Fifth Central Hospital of Tianjin (Tianjin, China) with 50% ± 5% humidity and 20–25°C ambient.

### 2.2. NSC Culture and Treatment

Rat NSCs were isolated and extracted from the hippocampus of new-born rats (within 1 day) under sterile conditions, digested with 0.05% trypsin for 15 minutes, and carefully pipetted with a dropper to form a single cell suspension at 1000 r/min. Trypsin was removed after centrifugation for 5 min. Neural stem cells were cultured in rat neural stem cell culture medium (Cyagen Biosciences, Suzhou, China). After 5-7 days of culture, the neurospheres were dissociated into single cell suspensions by mechanical separation for subculture, and the cells were seeded at a density of 2 × 10^5^ cells/. Cells of neurospheres were confirmed to be NSCs and propagated for 2 passages to obtain enough NSCs for experiments. Cultures maintained at 37°C and 5% CO_2_ in an incubator were recorded as the control group (Con). Hypoxia was performed by placing NSCs in 1% O_2_, 94% N_2_, 5% CO_2_, balanced nitrogen, and 95% humidity for 12 h (designated as H 12 h). For the mild hypothermia group, incubators were set at 33°C (designated as 33°C). All the experiments were carried out after a subsequent 48 h of culture under normal conditions.

### 2.3. Small Interfering RNA and Gene Transfection

For UBC9 knockdown, UBC9 siRNA (sc-36774) and nonsilencing control siRNA were purchased from Santa Cruz Biotechnology (Dallas, TX, USA, designated as siUBC9 and Con groups). Rat UBC9 cDNA was subcloned into the mammalian expression plasmid pcDNA3.1 (Life Technologies, Waltham, MA, USA), which containing a FLAG tag at the C-terminus (designated as UBC9 or NSC UBC9). siRNA and plasmids were electroporated into NSCs with a Nucleofector instrument (Lonza, Basel, Switzerland). UBC9-transfected NSCs were screened with neomycin (Sigma St. Louis, MO, USA).

### 2.4. Lactate Dehydrogenase (LDH) Detection, Flow Cytometry, and ECAR Detection

NSCs were collected by centrifugation of 100∗*g* for 5 min. LDH content in conditioned medium was detected using enzyme-linked immunosorbent assay (ELISA), based on the LDH Activity Assay Kit (Yuanmu Biotechnology Co., Ltd., Shanghai, China) and tested according to the product instructions. The percentage of apoptotic NSCs was determined by flow cytometry assay. After treatments, NSCs were harvested, washed, and then stained with fluorescein isothiocyanate- (FITC-) labeled annexin V and propidium iodide (PI) (Beyotime Biotechnology, Shanghai, China) in dark place for 5 min. After washing for 3 times with phosphate-buffered saline (PBS), percentages of apoptotic were quantified by flow cytometry (NovoCyte D2040R; Hangzhou, China). In addition, the extracellular acidification rates (ECAR) were detected using a Seahorse XF 96 Extracellular Flux Analyzer (Agilent Technologies, Santa Clara, CA, USA) according to instrument description.

### 2.5. Western Blot Analysis Assay

After extraction of protein from NSCs, the protein concentrations were determined by bicinchoninic acid assay (Thermo Fisher Scientific, Waltham, MA). Twenty micrograms protein of each sample in an equal volume was electrophoresed on 10%–12% polyacrylamide gels, before transfer onto a polyvinylidene fluoride membrane. After blocking the membrane in skim milk for 1 h, antibodies against SUMO1 (ab133352, 1 : 1000; Abcam, Cambridge, UK), SUMO2/3 (ab3742, 1 : 1000), UBC9 (ab75854, 1 : 1000), Oct4 (ab181557, 1 : 1000), SOX2 (ab92494, 1 : 1000), caspase-3 (ab184787, 1 : 1000), and glyceraldehyde-3-phosphate dehydrogenase (GAPDH; ab9485, 1 : 1000) were incubated overnight at 4°C. Then, the membranes were washed five times with TBST, followed by incubation with horseradish peroxidase-conjugated goat anti-rabbit IgG (111-035-003; 1 : 2,000; Jackson Immuno Research Laboratories, Inc., West Grove, PA, USA) antibody for 1 h at room temperature. GAPDH was used as internal control. Finally, membranes were exposed using ECL Plus substrate (Thermo Fisher Scientific, Waltham, MA). Data were evaluated by image analysis software (ImageJ version 1.48; National Institutes of Health, Bethesda, MD, USA).

### 2.6. Cell and Tissue Immunofluorescence

NSCs were mechanically dispersed and seeded on poly-L-lysine-coated coverslips in a 48-well cell culture plate. After being exposed to 4% paraformaldehyde for 15 min, NSCs were permeabilized with 0.2% Triton X-100 for 20 min and blocked with PBS containing 5% goat serum for another 30 min. Coverslips were incubated with antibodies against nestin (ab237036, 1 : 500) or Neuron-Specific Enolase (NSE; ab79757, 1 : 500) and Glial Fibrillary Acidic Protein (GFAP; ab279290, 1 : 500) overnight at 4°C. After washing for 4 times, mixtures of goat anti-mouse IgG H&L (AlexaFluor®488, ab150113, 1 : 200, Abcam) or goat anti-rabbit IgG H&L (AlexaFluor®594, ab150080, 1 : 200, Abcam) were dropped onto the coverslips. At last, nuclei were stained with 4′,6-diamidino-2-phenylindole (DAPI; Zhongshanjinqiao, Beijing, China) for 10 min. Images were acquired by a fluorescence microscope (Carl Zeiss, Oberkochen, Germany). For paraffin sections of rat brain tissues, the fixation, dehydration, embedding, sectioning, and dewaxing steps were added.

### 2.7. Establishment of Rat MCAO Models

A total number of 60 adult male Sprague-Dawley rats were randomly divided into 5 groups. During the operation, a small-animal ventilator (Shanghai Yuyan Instruments Co., Ltd., Shanghai, China) was used to maintain animals' respiration, and body temperature was monitored by a rectal temperature control. Making a 1 cm longitudinal incision between rat sternum and mandible, then left common carotid artery was isolated, and we found out the external carotid and internal carotid arteries under a stereo microscope (Olympus Corporation, Tokyo, Japan). Next, we ligated the distal heart end of the external carotid artery and the proximal heart end of the carotid artery, and a modified nylon thread (with 0.23 mm head diameter and 0.18 mm trunk diameter) was inserted from the carotid artery to the middle cerebral artery (~12.0 mm deep) and fixed with surgical line.

### 2.8. Mild Hypothermic Treatment

Rats which underwent surgery without thread insertion were defined as the “sham operation” group. NSCs or UBC9 NSCs were transplanted to the ischemic penumbra after the establishment of MCAO models as reported in literatures [17, 18]. To make mild hypothermia, MCAO rats injected with NSCs were placed on an insulation blanket (Shanghai Yuyan Instruments), and a rectal temperature monitor was to keep body temperature at 32 to 34°C for 12 h. Rats were then removed from blanket and gradually recovered to normal body temperature. After removal, some models' brains were stripped and sliced then incubated in 1% 2,3,5-triphenyl-2H-tetrazolium chloride (TTC, Sigma-Aldrich, St. Louis, MO) for 20 min at 37°C to distinguish the infarct area (white) and the uninfarct area (pink and red). Sections were fixed with 4% paraformaldehyde for 2 h to distinguish stained from unstained areas. The infarcted and uninfarcted areas were analyzed by ImageJ software (National Institutes of Health, Bethesda, MD), and percentages of infarct were calculated as (infarct area)/(area of the whole brain slice) × 100%. Brain tissues under the same conditions should be collected for paraffin section and immunofluorescence staining assay as described in Section 2.6.

### 2.9. Neural Function Analysis

Animals recovered from MCAO for 1, 4, 7, 14, 21, or 28 days before assess neurological functions by modified Neurological Severity Scores (mNSS) [19, 20]. The mNSS consisted of balance, movement, sensory function, and reflex tests with a score ranging from 0 to 18 (normal score: 0; maximum defect score: 18). In addition, rotarod testing was performed to evaluate of rat neurological deficits (Zhishuduobao Biotechnology Co., Ltd, Beijing, China). Rats were pretrained for 3 times before MCAO, and the experiment was performed for 7 days after MCAO. The cylinder accelerated from 10 to 40 rpm within 5 min; before rats fell from the rod, the latency to fall was recorded. Mean latency for each rat was calculated from three trials with a 30 min interval between 2 trials.

### 2.10. Rat Behavior Tests

7 days after MCAO, rats should be tested for behaviors. Spontaneous activity was monitored within 30 min for distance traveled and time spent in corners. Activity was assessed as distance traveled (locomotion), vertical activity (rearing), thigmotaxis, and time spent in corners using behavioral tester (Zhishuduobao Biotechnology Co., Ltd, Beijing, China) equipment. On the 10th day after MCAO, rats were tested for memory and learning abilities in the Morris water maze (Zhishuduobao Biotechnology Co., Ltd, Beijing, China) according to reference [21]. Rats underwent the visible platform experiment for the first 2 days, the nonvisible platform experiment for the following 3 days, and the probe trial for the last day. Escape latency and swimming paths were measured during the first 5 days. In the probe trial, percentages of time spent in quadrant IV and numbers of platform crossing were recorded.

### 2.11. Data Statistics and Analysis

Each experiment was performed at least for 3 times. Data are showed as mean ± standard deviation (SD) and were analyzed using GraphPad Prism 6 software (San Diego, CA). A *P* value <0.05 was considered significant difference. One-way ANOVA or the unpaired Student's *t* test was used to evaluate the significance of differences among treatment groups, as appropriate.

## 3. Results

### 3.1. Hypoxia Increased Injury, Inhibited Differentiation, Increased the Stemness Maintenance Potential, and Reduced the Metabolic Capacity of NSCs

After 12 h of hypoxia stimulation, the content of LDH released by NSCs increased significantly, suggesting cell damage (Figure 1(a)). The results showed that the percentage of apoptotic cells reached 30% after hypoxia (Figure 1(b)). Immunofluorescence detection showed that a certain proportion of NSCs spontaneously differentiated under normal conditions. NSE and GFAP were expressed. Nestin, a marker of NSCs, was highly expressed, and cells showed extensional growth morphology similar to nerve fiber structures. After hypoxia, NSCs exhibited obvious spherical growth, NSE and GFAP expression decreased, and nestin expression significantly increased (Figure 1(c)). Moreover, expression of stem cell markers Oct4 and SOX2 increased significantly (Figure 1(d)). Additionally, we calculated ECAR levels and found that hypoxia could significantly increase the anaerobic hydrolysis level of NSCs (Figure 1(e)).

### 3.2. Mild Hypothermia Antagonized Hypoxia-Induced Injury, Inhibited Differentiation, and Further Increased the Stemness Potential of NSCs

Mild hypothermia (33°C) significantly inhibited the damage induced by hypoxia at 37°C, significantly decreased the content of LDH, and reeducated the percentage of apoptotic cells to 20% (Figures 2(a) and 2(b)). Immunofluorescence detection showed that mild hypothermia significantly increased the expression of the NSC marker nestin and significantly reduced the expression of NSE and GFAP, and cells showed smooth nerve spherical growth (Figure 2(c)). Expression of Oct4 and SOX2 was also increased by mild hypothermia compared with cells at 37°C exposed to hypoxia (Figure 2(d)). Mild hypothermia could reduce the metabolic level of cells and inhibit hypoxia-induced increases of anaerobic fermentation (Figure 2(e)).

### 3.3. Hypoxia Increased Whole-Protein SUMOylation in NSCs and Mild Hypothermia further Strengthened SUMOylation Modification

Western blot was used to detect whole-cell levels of the SUMOylation modification under the conditions of hypoxia, mild hypothermia, and their superposition. The results showed that hypoxia and hypothermia could significantly promote the binding of SUMO1 and SUMO2/3 to target proteins and had a superposition effect; however, it had little effect on free SUMOs. Further detection of conjugating enzyme E2 (UBC9) showed that hypoxia could promote the expression of this protein (Figures 3(a)–3(c)).

### 3.4. Overexpression of UBC9 Could Increase the Stemness and Hypoxia Tolerance of NSCs

We transfected NSCs with a plasmid carrying the UBC9 gene sequence and screened clones with high expression of UBC9. Protein detection showed that SUMO1 and SUMO2/3 conjugates in UBC9-overexpressing NSCs were significantly increased, as were the contents of stemness maintenance molecules Oct4 and SOX2 (Figures 4(a)–4(c)). Immunofluorescence detection showed that UBC9 overexpression could significantly increase the expression of the NSC marker nestin and promote spherical growth of cells. Under hypoxia, expression of differentiation markers in NSCs was further reduced, nestin expression was increased, and the cell ball became smaller and round (Figure 4(d)). Compared with the Con group, NSCs overexpressing UBC9 exhibited decreased cell damage after hypoxia, but there was no significant damage to cells under normoxia (Figure 4(e)). Hypoxia activated the cleaved caspase-3 apoptosis signal in NSCs and promoted apoptosis, but UBC9 overexpression could partially reverse the proapoptotic damage induced by hypoxia (Figure 4(f)).

### 3.5. siUBC9 Reduced the Stemness and Hypoxia Tolerance of NSCs

We used small interfering RNA sequences to knockdown UBC9 expression. Protein detection showed that low UBC9 expression inhibited the modification of target proteins by SUMO1 and SUMO2/3 in NSCs, and expression of the stemness maintenance molecules Oct4 and SOX2 was significantly decreased (Figures 5(a)–5(c)). Immunofluorescence detection showed that low UBC9 expression could significantly inhibit nestin expression and promote cell differentiation. However, under hypoxic conditions, expression of differentiation markers in NSCs was further reduced, as was nestin expression, which may cause irreversible damage to NSCs (Figure 5(d)). Compared with the control group, NSCs with low UBC9 expression exhibited increased LDH release, which was further increased after hypoxia (Figure 5(e)). Low expression of UBC9 could activate the cleaved caspase-3-mediated apoptosis pathway in cells. Under hypoxia, cleaved caspase-3 activation further increased and promoted the expression of its precursor form (Figure 5(f)). Thus, low UBC9 expression significantly aggravated the hypoxic injury of NSCs.

### 3.6. Mild Hypothermia Increased the Survival of NSCs Transplanted into the Cerebral Ischemic Penumbra of Mice and Improved Neuromotor Function

MCAO could generate infarct areas reaching 50% in rats, and the infarct area could be reduced to 30% after transplantation of NSCs into the penumbra, while mild hypothermia could further reduce the infarct area. Immunofluorescence staining showed that NSC transplantation could significantly increase the density of NSCs in the penumbra, and mild hypothermia could further increase the survival of NSCs (Figures 6(a) and 6(b)). Compared with the MCAO group, the motor and coordination ability of rats transplanted with moderately hypothermic NSCs improved after 7 days (Figure 6(c)), and the neural function of rats significantly improved after 21 days (Table 1). Notably, postoperative MCAO rats showed anxiety, which was significantly relieved after NSC transplantation and mild hypothermia (Figures 6(d) and 6(e)). Morris water maze testing showed that the learning and memory function of rats transplanted with NSCs into the penumbra and treated with mild hypothermia improved to varying degrees compared with after MCAO (Figures 6(f)–6(h)).

MCAO rats were treated with NSCs and/or mild hypothermia as follows: Sham, sham operation; MCAO, MCAO model without treatment; MCAO+NSC, MCAO rats transplanted with NSCs; MCAO+NSC 33°C, MCAO rats transplanted NSCs kept at 32–34°C for 12 h; MCAO+NSC UBC9, MCAO rats transplanted with UBC9-overexpressing NSCs. Neurological scores were obtained at 1, 4, 7, 14, 21, and 28 days following surgery in each group. Data are expressed as mean ± SD (*n* = 7). ^#^*P* < 0.05 vs. MCAO and ^&^*P* < 0.05 vs. MCAO+NSC.

### 3.7. Transplanted NSCs Overexpressing UBC9 in the Cerebral Ischemic Penumbra of Rats Exhibited Higher Survival Rates and Enhanced Neuromotor Function

Compared with simple transplantation of NSCs, UBC9-overepxressing NSCS could reduce the cerebral infarction area of rats from 30% to 12%. Moreover, overexpression of UBC9 could promote the survival of NSCs, as well as their ability to adapt to hypoxic injury of brain (Figures 7(a) and 7(b)). Compared with the NSC-transplanted group, MCAO rats transplanted with NSCs overexpressing UBC9 exhibited significantly improved motor ability and neurological functions (Table 1, Figure 7(c)), reduced anxiety levels, and enhanced learning functions to varying degrees (Figures 7(d)–7(h)).

## 4. Discussion

In this study, we first examined the effect of hypoxia on NSCs. The results show that although hypoxia damaged NSCs, it increased their potential to maintain stemness, inhibited their neuronal differentiation, and reduced their metabolism. Further studies showed that mild hypothermia antagonized hypoxia-induced damage to NSCs, further inhibiting their differentiation and reducing cell metabolism. To evaluate whether the protective effect of mild hypothermia on NSCs was related to the SUMO modification of proteins, we examined the effect of mild hypothermia on the expression of SUMOs in NSCs. The results show that hypoxia increased global SUMO modifications of NSCs, both SUMO1 and SUMO2/3, and mild hypothermia further strengthened these trends. These results preliminarily validated our hypothesis that hypoxia can increase the hypoxia tolerance of NSCs by increasing global SUMOylation, and mild hypothermia can enhance neuroprotective effects by reinforcing this trend.

To evaluate whether global SUMOylation is indispensable to improving the hypoxia tolerance of NSCs, we next overexpressed and silenced the UBC9 gene (the only E2-binding enzyme in the SUMO modification reaction) [22] in NSCs and evaluated their hypoxia tolerance and stemness maintenance potential. The results show that *Ubc9* overexpression increased both the stemness potential of NSCs and their tolerance to hypoxia; in contrast, silencing UBC9 reduced the stemness of NSCs and decreased their tolerance to hypoxia. These results indicate that global SUMO modification of target proteins is essential to improve the tolerance of NSCs to hypoxia. However, we cannot specify exactly which proteins were SUMO-modified during this event. According to previous studies, we speculate that hypoxia greatly increases SUMO modification levels of numerous target proteins, including HIF-1*α*, Oct4, and SOX2. Theoretically, SUMO-modified HIF-1*α*, Oct4, and SOX2 cannot be degraded by ubiquitin hydrolase [23–25], thus allowing these proteins to persist and stably exist in the nucleus and cytoplasm of NSCs, whereby they increase hypoxia tolerance and stemness potential.

Finally, we established an MCAO model in rats to investigate the effects of mild hypothermia on survival of NSCs transplanted in the cerebral ischemic penumbra and subsequent improvements of neurological function. The results show that mild hypothermia increased the survival of NSCs transplanted in the cerebral ischemic penumbra of rats and improved their neurological functions, including motor and learning abilities. Finally, we transplanted NSCs overexpressing UBC9 into the cerebral ischemic penumbra of rats and found that these cells exhibited higher survival rates and better improved the neurological function of experimental animals, including motor and learning functions.

These results verify our hypothesis that increasing global SUMOylation of many target proteins, e.g., by overexpressing UBC9, can help NSCs obtain stronger hypoxia tolerance. Moreover, transplantation of NSCs with stronger hypoxia tolerance into the cerebral ischemic penumbra and subsequent mild hypothermia treatment increased the survival of NSCs in the penumbra and enhanced the neurological function of animals.

Although this study has enriched new ideas for the future treatment of ischemic cerebrovascular disease with mild hypothermia therapy combined with NSCs transplantation, there are still many difficult problems to be solved before it is actually applied to the clinic. First, due to the existence of the blood-brain barrier, how to inoculate NSCs into the brain of patients with cerebral ischemia will be a difficult problem for clinicians to face. Second, how to control the time window of hypothermia cooling and rewarming to produce the best therapeutic effect on patients is far from being interpreted. Third, the potential tumorigenic effects brought about by the proliferative characteristics of NSCs are serious side effects that we can never ignore. Last but not the final, SUMOylation can simultaneously intervene in the posttranslational modification of thousands of proteins. How to achieve advantages and avoid disadvantages at the molecular level and protein function will be a problem that researchers attach great importance to. In conclusion, there is still a long way to go before the clinical application of mild hypothermia combined with NSCs transplantation in the treatment of ischemic cerebrovascular disease.

## 5. Conclusions

Global protein SUMO modification is an important molecular mechanism for NSC tolerance of hypoxia, and mild hypothermia can further increase the degree of global protein SUMO modification in NSCs—a newly discovered molecular mechanism by which mild hypothermia protects the brain. Indeed, mild hypothermia can improve the hypoxia tolerance of NSCs and increase their survival following transplantation in situ, thus yielding better nerve repair effects.

## Figures and Tables

**Figure 1:** Effect of 12 h hypoxia on NSCs. (a) LDH contents of control and hypoxia groups were measured by ELISA. (b) Apoptosis was measured by flow cytometry of the two groups. Data shown indicate mean ± SD (*n* = 4). (c) Expression of NSE or nestin (red fluorescent signal) and GFAP (green fluorescent signal) in NSCs of the control and hypoxia groups was examined by immunofluorescence; DAPI (blue) was used to stain cell nuclei (scale bar, 20 *μ*m). (d) Oct4 and SOX2 protein expression was examined by western blotting. GAPDH was used for normalization. Data shown indicate mean ± SD (*n* = 3). (e) ECAR analysis of the glycolytic capacity of the control and hypoxic NSCs. Data shown indicate mean ± SD (*n* = 5); ^∗∗^*P* < 0.01 compared with the control group.

**Figure 2:** Effect of mild hypothermia (33°C) on hypoxic NSCs. (a) LDH contents of the control (37°C) and mild hypothermia groups were measured by ELISA. (b) Apoptosis assays were measured by flow cytometry. Data indicate mean ± SD (*n* = 4). (c) Expression of NSE or nestin (red fluorescent signal) and GFAP (green fluorescent signal) in the control NSCs or mildly hypothermic and hypoxic NSCs was examined by immunofluorescence; DAPI (blue) was used to stain cell nuclei (scale bar, 10 *μ*m). (d) Oct4 and SOX2 protein expression was examined by western blotting. Data shown indicate mean ± SD (*n* = 3). (e) ECAR analysis of the glycolytic capacity of the control NSCs or mildly hypothermic and hypoxic NSCs. Data shown indicate mean ± SD (*n* = 5); ^∗^*P* < 0.05 and ^∗∗^*P* < 0.01 compared with 37°C group.

**Figure 3:** Effects of hypoxia (H 12 h) and mild hypothermia (33°C) on whole-protein SUMO modification in NSCs. (a) and (b) Expression of SUMO1 and SUMO2/3 conjugates, free SUMO1 and SUMO2/3, and UBC9 in NSCs after hypoxia and/or moderate hypothermic treatment, as assessed by western blotting. (c) Quantitative data were normalized to GAPDH and are expressed as mean ± SD (*n* = 3). ^∗^*P* < 0.05, ^∗∗^*P* < 0.01, and ^∗∗∗^*P* < 0.001 vs. control.

**Figure 4:** Overexpression of UBC9 increased NSC stemness and tolerance to hypoxia. (a) and (b) Expression of SUMO1 and SUMO2/3 conjugates, free SUMO1 and SUMO2/3, UBC9, Oct4, and SOX2 in NSCs overexpressing UBC9, as assessed by western blotting. (c) Quantitative data were normalized to GAPDH and expressed as mean ± SD (*n* = 3). (d) Expression of NSE or nestin (red fluorescent signal) and GFAP (green fluorescent signal) in NSCs of the UBC9 transgene and Con groups after 12 h hypoxia was examined by immunofluorescence; DAPI (blue) was used to stain cell nuclei (scale bar, 10 *μ*m). (e) LDH contents were measured by ELISA, and data shown indicate mean ± SD (*n* = 4). (f) Western blotting to detect cleaved caspase-3 expression in NSCs. Quantitative analysis: cleaved caspase-3 expression was normalized to GAPDH and is expressed as mean ± SD (*n* = 3). ^∗^*P* < 0.05 and ^∗∗^*P* < 0.01 vs. control.

**Figure 5:** UBC9 interference reduced NSC stemness and tolerance to hypoxia. (a) and (b) Expression of SUMO1 and SUMO2/3 conjugates, free SUMO1 and SUMO2/3, UBC9, Oct4, and SOX2 in NSCs after UBC9 interference. (c) Quantitative data were normalized to GAPDH and are shown as mean ± SD (*n* = 3). (d) Expression of NSE or nestin (red fluorescent signal) and GFAP (green fluorescent signal) in NSCs of the siUBC9 or Con groups after 12 h hypoxia was examined by immunofluorescence; DAPI (blue) was used to stain cell nuclei (scale bar, 10 *μ*m). (e) LDH contents were measured by ELISA, and data shown indicate mean ± SD (*n* = 4). (f) Western blotting to detect the expression of cleaved caspase-3 in NSCs. Quantitative analysis: cleaved caspase-3 expression was normalized to GAPDH and is expressed as mean ± SD (*n* = 3). ^∗^*P* < 0.05 and ^∗∗^*P* < 0.01 vs. control.

**Figure 6:** Mild hypothermia increased the survival of NSCs transplanted into the ischemic penumbra of rats and improved neuromotor function.(a) Representative TTC-stained coronal brain sections of sham-operated (Sham) rats, MCAO rats, MCAO rats transplanted with NSCs (MCAO+NSC), and MCAO rats transplanted with NSCs kept at 32–34°C for 12 h (MCAO+NSC 33°C). Immunofluorescence staining of cerebral cortex tissue sections (scale bar, 20 *μ*m). (b) Quantification of percentages of cerebral infarct volume (*n* = 5) and proportions of nestin-positive to DAPI-positive cells (*n* = 4); data are expressed as mean ± SD. (c) Rotarod testing was used to analyze the neurological deficits of rats in each group. (d) Spontaneous activity in the open field over30 min and (e) time spent in corners. (f)–(h) Escape latency to find the nonvisible platform. Number of crosses in the probe test and time spent in quadrant IV. Data shown indicate mean ± SD (*n* = 7). ^∗^*P* < 0.05 and ^∗∗^*P* < 0.01 vs. Sham, ^#^*P* < 0.05 and ^##^*P* < 0.01 vs. MCAO.

**Figure 7:** UBC9 overexpression increased the survival of NSCs transplanted into the ischemic penumbra of rats and improved neuromotor function. (a) Representative TTC-stained coronal brain sections of MCAO+NSC and MCAO rats transplanted with UBC9-overexpressing NSC (MCAO+NSC UBC9) groups. Immunofluorescence staining of cerebral cortex tissue sections (scale bar, 20 *μ*m). (b) Quantification of percentages of cerebral infarct volume (*n* = 5) and proportions of nestin-positive to DAPI-positive cells (*n* = 4), and data are expressed as mean ± SD. (c) Rotarod testing was used to analyze the neurological deficits of rats in each group. (d) Spontaneous activity in the open field over 30 min and (e) time spent in corners. (f)–(h) Escape latency to find the nonvisible platform. Number of crosses in the probe test and time spent in quadrant IV. Data shown indicate mean ± SD (*n* = 7). ^∗^*P* < 0.05 vs. MCAO+NSC.

**Table 1:** Modified Neurological Severity Score (mNSS) results according to the time after MCAO.

mNSS scores	*n*	1 d	4 d	7 d	14 d	21 d	28 d
Sham	7	0.57 ± 0.79	0.43 ± 0.53	0.57 ± 0.53	0.43 ± 0.53	0.43 ± 0.53	0.71 ± 0.76
MCAO	7	12.29 ± 0.95	10.71 ± 0.76	9.14 ± 0.90	7.86 ± 0.69	7.17 ± 0.75	6.14 ± 0.90
MCAO+NSC	7	12.29 ± 1.11	10.29 ± 0.95	8.29 ± 0.95	6.43 ± 0.53	5.43 ± 0.98	4.29 ± 0.95
MCAO+NSC 33°C	7	12.14 ± 1.46	10.57 ± 1.40	7.43 ± 1.40	5.74 ± 2.00	3.29 ± 0.76^#^	2.29 ± 0.76^#&^
MCAO+NSC UBC9	7	11.43 ± 0.79	10.14 ± 1.07	9.86 ± 3.48	4.29 ± 0.76^#^	2.86 ± 0.69^#&^	2.43 ± 0.98^#&^

## Data Availability

All the data used to support the findings of this study are available from the corresponding authors upon request.
